The article "Optimized extraction, composition, antioxidant and antimicrobial activities of exo and intracellular polysaccharides from submerged culture of Cordyceps cicadae" was retracted in 2018. Reasons: duplicated images; concerns about the data.

# Optimized extraction, composition, antioxidant and antimicrobial activities of exo and intracellular polysaccharides from submerged culture of *Cordyceps cicadae*

**DOI:** 10.1186/s12906-015-0967-y

**Published:** 2015-12-23

**Authors:** Sapan Kumar Sharma, Nandini Gautam, Narender Singh Atri

**Affiliations:** Department of Plant Pathology, CSK, Himachal Pradesh Agriculture University, Palampur, (176 062) India; Centre for Environment Science and Technology, School of Environmental and Earth Sciences, Central University of Punjab, Bathinda, (151 001) India; Department of Botany, Punjabi University Patiala, Punjab, (147 002) India

**Keywords:** *Cordyceps cicadae*, EPS, IPS, Antioxidant, Monosaccharides, Antimicrobial activity

## Abstract

**Background:**

*Cordyceps cicadae* is known as Jin Chan Hua in Traditional Chinese Medicine and known to possess different pharmacological activities. Presently, it was collected from the wild and isolated. Mycelial culture was optimized for extraction of polysaccharides under submerged culture conditions. Besides antioxidant, antibacterial activities of extracted polysaccharides were tested for first time.

**Methods:**

Exo-polysaccharides (EPS) and intracellular polysaccharides (IPS) production was tested under different factors (medium capacity, rotation speed, pH, incubation time, temperature, carbon, nitrogen, minerals sources and carbon to nitrogen ratio) by orthogonal experiments using one-factor-at-a-time method. Monosaccharides composition of polysaccharides produced by *C. cicadae* was determined using high performance liquid chromatography. Antioxidant and antimicrobial activities on eight bacterial strains were checked by different standard procedures.

**Results:**

Factors viz., medium capacity, rotation speed, incubation time, pH and temperature affected the EPS and IPS production under submerged culture conditions. EPS and IPS production was observed to vary with different carbon and nitrogen sources as well as C/N ratio. Glucose was the major component of polysaccharides (63.10 ± 4.15 %). Extracted EPS and IPS showed higher antioxidant potential with significant DPPH radical scavenging activity, ABTS radical scavenging activity, reducing power and iron chelating activity. Antimicrobial activities of EPS and IPS varied among the tested bacterial strains. IPS showed slightly higher inhibition rate to all the tested bacterial strains as compared to EPS. Maximum inhibition zones of IPS (12.9 ± 0.2 mm) and EPS (12.5 ± 0.3 mm) was observed against *Pseudomonas aeruginosa* at 10 % con. However, both EPS and IPS fractions showed broad spectrum for all the pathogenic microbial strains tested. The MIC of both the extracts ranged from 60–100 mg/mL.

The article "Optimized extraction, composition, antioxidant and antimicrobial activities of exo and intracellular polysaccharides from submerged culture of Cordyceps cicadae" was retracted in 2018. Reasons: duplicated images; concerns about the data.

**Conclusions:**

EPS and IPS production from submerged culture of *C. cicadae* with significant antioxidant and antibacterial potential can be enhanced with the combination of several factors which can be used for large scale industrial fermentation of *C. cicadae*.

## Background

*Cordyceps* is a widely distributed genus with more than 400 species worldwide [1–3]. Species of *Cordyceps* are known as the source of disease combating natural product with tremendous biological activities. Extracts from the fruit bodies and mycelium of this fungus exhibit different pharmacological activities [4]. Species like *Cordyceps sinensis* has been used extensively to cure various cancerous diseases and known to possess immunomodulatory activities [5–9]. The range of polysaccharides present in *Cordyceps* mycelium ranges 3–8 % and are the main constituents [10–12]. *Cordyceps* species are the sources of several bioactive constituents like cordycepin and others which possess liver protective effects, antioxidative activities, enhances the T-cell and macrophages activity, reduce the level of c-Myc, c-Fos, and VEGF levels in the lungs and liver by exopolysaccharide fraction, and reduce the level of cholesterol and triglyceride [13–16]. Beside, some uncommon cyclic dipeptides, including co- cyclo-[Gly-Pro], cyclo-[Leu-Pro], cyclo-[Val-Pro], cyclo-[Ala-Leu], cyclo-[Ala-Val], and cyclo-[Thr-Leu] and small amounts of polyamines, such as 1,3-diamino propane, cadaverine, spermidine, spermine, and putrescine are also extracted from these which exhibit multiple pharmacological activities including antitumor, anti-inflammatory, mmunopotentiation, hypoglycemic, and hypocholesterolemic effects, protection of neuronal cells against the free radical-induced cellular toxicity, steroidogenesis, and antioxidant activities [17–20].

*Cordyceps cicadae* is known as Jin Chan Hua in Traditional Chienese Medicine and the extract from this species is used against kidney diseases, immune related diseases, and cancer [21–23]. Extracts from *C. cicadae* exhibit immuno-regulatory effects on human T lymphocytes and modulate the growth of mononuclear cells and also known to inhibit the growth of lung adeno-carcinoma and melanoma *in vivo* and *in vitro* [24–27].

EPS as well as IPS extracted from submerged culture of many *Cordyceps* species exhibited significant antioxidant and antimicrobial activities [28]. The productivity of polysaccharides has been found to vary with environmental conditions and medium composition, including carbon source, nitrogen source, and pH [29]. To add the medicinal potential and large scale industrial fermentation of *C. cicadae*, present studies were conducted to optimize the antioxidant EPS and IPS production by one-factor-at-a-time method and orthogonal matrix design. Monosaccharide composition, antioxidant and antimicrobial activities of EPS and IPS were also evaluated under present experiments.

The article "Optimized extraction, composition, antioxidant and antimicrobial activities of exo and intracellular polysaccharides from submerged culture of Cordyceps cicadae" was retracted in 2018. Reasons: duplicated images; concerns about the data.

## Methods

### Culturing and optimized extraction of polysaccharides

*Cordyceps cicadae* was collected from the sub-Himalayan forest at Macleodgang (Dharamshala, India) geographically located at 32.238602°N 76.323878°E, and identified through microscopical taxonomy, and ITS region sequencing and deposited at Herbarium, Department of Botany, Punjabi University, Patiala (PUN 7194) (Fig. 1a, b). Isolation was done on potato dextrose agar (PDA) slants. The slants were incubated at 25 °C for 10 days. Sub-culturing was done in every 30-days interval to maintain the viability. Submerged culturing was done in a standard basal medium (sucrose 30.0 g/L, yeast powder 5.0 g/L, peptone 5.0 g/L, MgSO4. 7H2O 1.0 g/L, and KH2PO4 0.5 g/L) [30–32]. Effect of medium capacity (50, 100, 150, 200, and 250 mL), rotation speed (50, 100, 125, 150, 175, and 200 rpm) of culture medium, incubation time (2–10 days), pH (3.0–8.0), temperature (20, 23, 25, 27, 30, and 33 °C), carbon sources (glucose, galactose, sucrose, mannitol, maltose, and fructose), nitrogen sources (yeast extract, peptone, NaNO2 (NH4)2SO4, and L-arginine HCL), mineral sources (CaCl2, CoCl2.6H2O, FeSO4.7H2O, KH2PO4, K2HPO4, MnCl2.6H2O) and C/N (1 : 5, 1 : 10, 1 : 20, 1 : 30, and 1 : 40) ratio on EPS and IPS production was studied by orthogonal experiments using one-factor-at-a-time method.

**Fig. 1:** **a** Wild fruitbody of *C. cicadae,* **b** 6 days old mycelium, **c** DPPH scavenging activity of EPS and IPS, **d** ABTS radical scavenging activity of EPS and IPS, **e** Reducing power of EPS and IPS, **f** Iron chelating activity of EPS and IPS

### Extraction of polysaccharides

Exo-polysaccharides (EPS) were extracted by the standard method with some modifications [33]. For this, mycelial biomass in the medium was centrifuged at 10,000 × g for 10 min. The supernatant obtained was mixed with three volumes of pure ethanol and left for 24 h at 4 °C. The resulting precipitate was then separated by centrifugation at 8000 × g for 10 min. The precipitate (EPS) was washed with ultrapure water and subsequently lyophilized for quantitative assessment and analysis.

For intracellular polysaccharides, mycelial biomass was subjected to extraction with boiling water for an hour and the mixture was filtered through Whatman number 1 filter paper. The filtrate was allowed to precipitate with four volumes of 95 % (v/v) ethanol and left overnight at 4 °C. Precipitates obtained were separated by centrifugation at 8000 × g for 10 min. The precipitates (IPS) were washed with ultrapure water and subsequently lyophilized for quantitative assessment and analysis [34].

The article "Optimized extraction, composition, antioxidant and antimicrobial activities of exo and intracellular polysaccharides from submerged culture of Cordyceps cicadae" was retracted in 2018. Reasons: duplicated images; concerns about the data.

### Monosaccharide composition

Monosaccharide composition of polysaccharides was determined by high performance liquid chromatography coupled to an evaporative light scattering detector [35]. Polysaccharide fraction (0.1 g) was extracted with 2.5 mL of 70 % aqueous methanol followed by 1.5 mL of 70 % aqueous methanol and then 1 mL of 70 % aqueous methanol. This extract was centrifuged at 4000 rpm at 4 °C for 10 min. Supernatant was collected and volume made up to 5 mL with 70 % methanol. The extract was passed through Millipore filter (0.45 m) prior to injection on the HPLC.

### DPPH radical scavenging activity

The DPPH scavenging activity was measured by the standard method described by Emanuel [36]. Briefly, DPPH (200 μm) solution at different concentrations (2–10 mg/mL) was added to 0.05 mL of the samples dissolved in ethanol. An equal amount of ethanol was added to the control. Ascorbic acid was used as the control. The absorbance was read after 20 min., at 517 nm and the inhibition was calculated using the formula:

DPPH scavenging effect (%) = A0-AP/A0 × 100, where A0 was the absorbance of the control and AP was the absorbance in the presence of the sample.

### ABTS radical scavenging assay

ABTS radical scavenging activity was measured by method described by [37]. For this, 10 μL of the sample was added to 4 mL of the diluted ABTS^*•*+^ solution (prepared by adding 7 mM of the ABTS stock solution to 2.45 mM potassium persulfate, kept in the dark, at room temperature, for 12–16 h before use). The solution was then diluted with 5 mM phosphate-buffered saline (pH 7.4). The absorbance was measured after 30 min at 730 nm. Ascorbic acid was used as control. The ABTS radical-scavenging activity was calculated as

$$ Scavenging\  activity\left(S\%\right)=\left( Acontrol- Asample/ Acontrol\right)\times 100 $$

### Reducing power

Reducing power was estimated by standard method [38]. Briefly, 200 μL of the samples were mixed with sodium phosphate buffer (pH 6.6), 1 mM FeSO4, and 1 % potassium ferricyanide and incubated for 20 min at 50 *°*C after that trichloroacetic acid was added and the mixtures were centrifuged. Supernatant (2.5 mL) was mixed with an equal volume of water and 0.5 mL 0.1 % FeCl3. The absorbance was measured at 700 nm.

### Ferrous ion chelating assay

For this, 1 mL of the sample (2–10 mg/mL) was mixed with 3.7 mL of ultrapure water, following which the mixture was reacted with ferrous chloride (2 mmol/L, 0.1 mL) and ferrozine (5 mmol/L, 0.2 mL) for 20 min. and the absorbance was read at 562 nm. EDTA was used as positive control. The chelating activity on the ferrous ion was calculated using the formula: chelating activity (%) *=* [(Ab – As)/Ab] *×* 100, where Ab is the absorbance of the blank and As is the absorbance in the presence of the extract [39].

The article "Optimized extraction, composition, antioxidant and antimicrobial activities of exo and intracellular polysaccharides from submerged culture of Cordyceps cicadae" was retracted in 2018. Reasons: duplicated images; concerns about the data.

### Antimicrobial activities

EPS and IPS fractions were obtained as the method described above. Minimal inhibitory concentration (MIC) of the polysaccharide fractions were tested for *Escherichia coli*, *Klebsiella pneumonia, Vivrio cholerae*, *Pseudomonas aeruginosa*, *Vibrio alginolyticus*, *Staphylococcus aureus*, *Vibrio parahaemolyticus* and *Streptococcus pneumonia*. For this, bacterial strains were individually inoculated in the nutrient broth and incubated at 37 °C for 24 h. Mueller Hinton agar (MHA) is prepared and autoclaved and poured in petriplates and incubated at 37 °C for 24 h. The 24 h old bacterial broth cultures were inoculated in the petridishes. The stock solution of polysaccharides was prepared at a concentration of 100 mg/mL. Sterile antimicrobial disc was impregnated with polysaccharide of the four concentrations tested. Positive control disc containing tetracycline (1 mg/mL) and negative control as EDTA. These impregnated discs were allowed to dry at laminar air flow chamber for 2 h, and were placed at the respective bacterial plates and incubated at 37 °C for 24 h. The diameter (mm) of the growth inhibition halos produced by the polysaccharides was examined. Result was calculated by measuring the zone of inhibition in millimetres (mm). All the tests were performed in triplicate [40].

### Experimental design

For optimized extraction, different factors considered for the design were carbon sources, nitrogen sources, and ratio of carbon to nitrogen sources, temperature, pH value, medium capacities, rotation speed and culture time. According to the results of the single factor experiment, the orthogonal L9 (3^4^) was used for optimal culture conditions in submerged cultures.

The data were analyzed by one-way analysis of variance (ANOVA) using SPSS-16 version software. *p* values at <0.05 were considered for describing the significant levels.

## Results and discussion

### Optimized extraction of polysaccharide and monosaccharide composition

For optimized extraction of EPS and IPS, *Cordyceps cicadae* culture was grown in media with different medium capacities. The maximum EPS (455.19 ± 2.21 mg/L) and IPS (276.16 ± 2.10 mg/L) production was observed in 200 mL of the liquid medium, while least values of EPS (312.14 ± 2.41 mg/L) and IPS (111.23 ± 2.47 mg/mL) production were obtained in 50 mL of the medium. However, no significant difference (*p* < 0.05 %) were observed in EPS and IPS production in the medium capacities from 150 to 250 mL. Rotation speed showed direct relation with EPS and IPS production. Results obtained for effect of rotation speed on polysaccharide production showed maximum EPS (282.10 ± 1.99 mg/mL) and IPS (199.14 ± 1.66 mg/L) production in culture rotation speed 175 rpm. These results obtained showed variation in polysaccharide production. This variation is due to the fact of low oxygen requirement by the culture as shown in *C. ophioglossoides* and other ascomycetes [31, 41]. However, in the submerged culture of *C. ophioglossoides* maximum values for IPS production was obtained in 150 mL of medium with rotation speed 150 rpm [31]. Culture incubation time and pH range showed significant effect on EPS and IPS production. Mycelial culture of *C. cicadae* incubated for 6 days and pH 6.0 showed maximum EPS and IPS production (Table 1). In other medicinal species viz., *C. ophioglossoides* and *C. sinensis,* incubation period of 5–6 days and slightly acidic pH 5.0–6.0 promoted maximum IPS production [31, 42]. Favourable temperature for the production of EPS and IPS was found to be 23 °C. The findings obtained for the production of EPS and IPS are similar as obtained for *C. gracilis* culture [32]. However, this temperature for *C. sinensis* was observed as 20 °C and 25 °C for *C. ophioglossoides* [43].

The article "Optimized extraction, composition, antioxidant and antimicrobial activities of exo and intracellular polysaccharides from submerged culture of Cordyceps cicadae" was retracted in 2018. Reasons: duplicated images; concerns about the data.

**Table 1:** Effect of different factors on polysaccharides (EPS and IPS) yield in submerged culture of *C. cicadae*

Sources	EPS (mg/L)	IPS (mg/L)
Medium capacity/ml		
50	312.14 ± 2.41^c^	111.23 ± 2.47^a^
100	350.18 ± 2.41^d^	193.13 ± 2.12^b^
150	410.11 ± 4.68^d^	234.61 ± 2.11^b^
200	455.19 ± 2.21^e^	276.16 ± 2.10^c^
250	413.14 ± 2.17^d^	229.13 ± 1.41^a^
Rotation speed (rpm)		
50	211.14 ± 1.52^b^	110.11 ± 1.15^a^
100	239.12 ± 1.16^b^	134.12 ± 2.16^a^
125	268.15 ± 1.51^b^	152.21 ± 2.21^a^
150	274.11 ± 2.12^c^	192.10 ± 2.09 ^b^
175	282.10 ± 1.99^b^	199.14 ± 1.66^b^
200	172.19 ± 1.26^a^	175.21 ± 1.21^a^
Incubation time/d		
2	187.12 ± 1.26^b^	111.10 ± 1.49^a^
3	215.21 ± 1.27^b^	135.11 ± 2.12^a^
4	234.10 ± 1.18^c^	164.16 ± 1.92^a^
5	265.12 ± 1.79^c^	176.17 ± 1.42^a^
6	315.20 ± 2.15^d^	213.67 ± 2.11^b^
7	301.17 ± 2.10^c^	204.51 ± 1.98^a^
8	213.11 ± 2.43^b^	167.19 ± 1.46^a^
9	215.26 ± 1.91^b^	142.15 ± 1.91^a^
10	192.11 ± 2.63^b^	138.32 ± 2.12^a^
pH		
3.0	221.13 ± 2.12^c^	124.21 ± 1.25^a^
4.0	243.24 ± 2.99^c^	143.11 ± 1.26^a^
5.0	257.22 ± 1.35^c^	182.12 ± 1.39^a^
6.0	274.11 ± 2.52^c^	201.19 ± 1.60^b^
7.0	253.31 ± 2.44^c^	192.59 ± 1.26^a^
8.0	231.10 ± 1.12^b^	171.10 ± 1.33^a^
Temperature		
20	312.18 ± 2.95^c^	172.63 ± 2.33^a^
23	395.29 ± 2.16^d^	215.60 ± 1.71^b^
25	390.81 ± 2.55^c^	162.42 ± 2.62^a^
27	243.23 ± 3.41^b^	159.49 ± 1.46^a^
30	212.20 ± 2.90^b^	147.22 ± 1.91^a^
33	93.19 ± 2.61^a^	063.10 ± 2.46^a^

Values are expressed as mean ± SE and the same alphabets in the same column are not statistically significant according to Tukey’s test for multiple comparisons with < 0.05 for different conditions as mentioned in the table

Six different carbon sources were studies to find the suitable medium source for the production of EPS and IPS in *Cordyceps cicadae*. Although, all the tested carbon sources yielded EPS and IPS, but maximum EPS (354.22 ± 1.62 mg/L) and IPS (214.40 ± 2.18 mg/L) production took place in the medium supplemented with glucose. Glucose was found to be the best carbon source for mycelial culture growth in many medicinal *Cordyceps* sp. viz., *C. gracilis* [32], *C. ophioglossoides*, *C. militaris* and *C. sinensis* [44, 45]. Six different nitrogen sources were tested for maximum EPS and IPS production. Amongst them, peptone promoted maximum EPS (424.82 ± 2.39 mg/L) and IPS (264.19 ± 2.92 mg/L) production. Nitrogen requirement for mycelial growth is different in different species. Yeast extract was observed as the best nitrogen source for biologically active EPS and IPS of *C. gracilis* and other species of this genus [32, 43]. Six different mineral sources were tested to obtain maximum EPS and IPS production. Submerged culture of this medicinal fungus promoted maximum EPS (313.31 ± 2.49 mg/mL) and IPS (187.10 ± 2.36 mg/mL) production with KH2PO4 as mineral source. This mineral source also observed as the best mineral source for two medicinal *Cordyceps* sp. viz, *C. militaris* and *C. sinensis* [43]. C/N ratio 10:1 promoted maximum EPS (295.17 ± 2.15 mg/L) and IPS (232.11 ± 2.45 mg/L) production for *C. cicadae* (Table 2). Present results are in conformity with previous reports on *C. gracilis* and *C. ophiogllosoides*, as C/N ratio 10:1 provided maximum IPS (653.79 ± 5.24 mg/L) production [31, 32] [Table 2].

The article "Optimized extraction, composition, antioxidant and antimicrobial activities of exo and intracellular polysaccharides from submerged culture of Cordyceps cicadae" was retracted in 2018. Reasons: duplicated images; concerns about the data.

**Table 2:** Effect of different carbon and nitrogen sources on EPS and IPS yield in submerged culture of *C. cicadae*

Factors	EPS (mg/L)	IPS (mg/L)
Carbon sources		
Mannitol	302.26 ± 3.82^c^	144.71 ± 1.92^a^
Galactose	213.10 ± 2.29^c^	141.13 ± 1.46^a^
Sucrose	335.12 ± 2.81^c^	209.10 ± 2.11^b^
Glucose	354.22 ± 1.62^d^	214.40 ± 2.18^b^
Maltose	247.19 ± 1.48^b^	144.46 ± 1.46^a^
Fructose	211.34 ± 1.19^b^	142.20 ± 2.31^a^
Nitrogen source		
Yeast Extract	365.21 ± 3.82^d^	215.16 ± 3.74^b^
Peptone	424.82 ± 2.39^c^	264.19 ± 2.92^a^
NaNO_2_	305.17 ± 2.12^c^	148.15 ± 2.79^a^
(NH_4_)_2_SO_4_	293.14 ± 2.15^c^	124.12 ± 2.65^a^
L – Arginine HCL	254.33 ± 2.13^b^	99.49 ± 2.16^a^
DL – Ascorbic Acid	206.19 ± 1.98^b^	92.22 ± 2.11^a^
Mineral Sources		
CaCl_2_	231.17 ± 2.79^c^	116.63 ± 2.12^a^
CoCl_2_.6H_2_O	242.16 ± 2.45^d^	123.62 ± 1.98^b^
FeSO_4_.7H_2_O	264.13 ± 1.11^c^	144.42 ± 2.09^a^
KH_2_PO_4_	313.31 ± 2.49^b^	187.10 ± 2.36^a^
K_2_HPO_4_	275.21 ± 2.13^b^	162.32 ± 2.18^a^
MnCl_2_.6H_2_O	210.26 ± 1.92^b^	112.83 ± 2.90^a^
C/N ratio		
40:1	111.15 ± 2.07^a^	92.12 ± 2.13^a^
30:1	229.18 ± 2.32^c^	142.16 ± 2.57^a^
20:1	243.94 ± 2.79^c^	179.15 ± 2.36^a^
10:1	295.17 ± 2.15^c^	232.11 ± 2.45^b^
5:1	274.17 ± 2.91^c^	209.40 ± 1.99^b^
1:1	253.19 ± 2.64^c^	185.16 ± 2.37^a^

Values are expressed as mean ± SE and the same alphabets in the same column are not statistically significant according to Tukey’s test for multiple comparisons with < 0.05 for different conditions as mentioned in the table

Glucose was observed as the major monosaccharide in *C. cicadae* (63.10 ± 4.15 %) followed by rhamnose (39.11 ± 3.57 %), xylose (20.12 ± 2.29 %), mannose (15.16 ± 1.34 %), arabinose (2.05 ± 0.37 %), galactose (0.12 ± 0.0 %) and galacturonic acid (0.06 ± 0.0 %) (Table 3). Similar results were obtained for polysaccharide composition of *C. gracilis*, *C. militaris* and other medicinal basidiomycetes, in which glucose was found to be the major monosaccharide along with sucrose and galactose [32, 36, 46]. Results obtained for effect of different factors on yield of EPS and IPS showed a significant effect. Results revealed the effect on EPS and IPS production in the order as: temperature > incubation time > pH > rotary speed > medium capacity (Table 4).

**Table 3:** Monosaccharide composition of polysaccharides in *C. cicadae*

Monosaccharides	(%)
Xylose	20.12 ± 2.29
Glucose	63.10 ± 4.15
Rhamnose	39.11 ± 3.57
Mannose	15.16 ± 1.34
Arabinose	2.05 ± 0.37
Galacturonic acid	0.06 ± 0.0
Galactose	0.12 ± 0.0

**Table 4:** Results obtained for orthogonal design by one factor at a time method

Experimental group	Temperature (°C)	pH	Rotary speed/r · min − 1	Culture time/d	EPS (mg/L)	IPS (mg/L)
1	1	1	1	1	312.13 ± 1.75	262.81 ± 2.60
2	1	2	2	2	367.10 ± 12.19	310.12 ± 11.26
3	1	3	3	3	377.15 ± 12.19	334.21 ± 12.29
4	2	1	2	3	598.41 ± 22.10	378.12 ± 24.10
5	2	2	3	1	564.68 ± 13.19	401.56 ± 12.19
6	2	3	1	2	648.69 ± 9.18	421.60 ± 6.77
7	3	1	3	2	238.15 ± 42.17	188.10 ± 12.27
8	3	2	1	3	364.15 ± 3.79	250.10 ± 2.70
9	3	3	2	1	209.16 ± 28.11	166.16 ± 15.7
K_1_	10.16	9.18	14.84	14.65		
K_2_	22.11	13.91	13.78	14.98		
K_3_	11.15	9.02	14.06	14.39		
R	12.10	4.15	0.82	2.19		
K_1_*	452.16	343.80	422.13	317.46		
K_2_*	572.19	516.12	542.14	378.16		
K_3_*	312.18	318.10	362.18	412.21		
R*	382.11	82.18	23.18	97.75		

K_1_ = Σ EPS at culture factor level1/3., K_1_* = Σ IPS yield at culture factor level1/3

The article "Optimized extraction, composition, antioxidant and antimicrobial activities of exo and intracellular polysaccharides from submerged culture of Cordyceps cicadae" was retracted in 2018. Reasons: duplicated images; concerns about the data.

### Antioxidant and antimicrobial activities of EPS and IPS

The DPPH scavenging activity of EPS and IPS extracted from the mycelium of *C. cicadae* showed positive direct correlation with the concentration of the sample (Fig. 1c). EPS and IPS extracted from *C. cicadae* showed high DPPH scavenging activity. The results are also supported by EC50 values, which were found to 7*.*32 ± 0*.*09 mg/mL for EPS and 6*.*79 ± 0*.*04 mg/mL for IPS (Table 5). High DPPH scavenging activities of EPS and IPS are similar to other medicinal species like *C. gracilis*, *C. militaris* and *C. sinensis* [32, 47, 48]. The inhibition percentage of the ABTS radical by EPS and IPS of *C. cicadae* was found to be directly depended upon the concentration of the sample. The scavenging effect of all the extracts increased with increasing concentration as shown in the figure. At a concentration of 8.0 mg/mL, the percentage inhibition of EPS and IPS were found to be the maximum. High concentrations of the EPS and IPS are able to quench the free radicals in the system. The results indicated that the EPS and IPS of *C. cicadae* possessed significant scavenging power for the ABTS radicals (Fig. 1d). The results obtained for reducing power abilities of EPS and IPS in submerged culture of *C. cicadae* showed that both types of polysaccharides possessed the reducing capacity. The reducing powers of EPS and IPS increased as the concentration increased (Fig. 1e). The reducing power of IPS was found to be higher than reducing power of EPS and at concentration 8 mg/mL maximum difference in the reducing power of IPS (0.53 ± 0.02 mg/mL) and EPS (0.42 ± 0.00 mg/mL) was observed. The reducing power of polysaccharides is due to presence of reductones and present results showed that EPS and IPS of *C. cicadae* contained reductones which react with precursors of peroxides to prevent peroxide formation [32]. The iron chelating ability of the EPS and IPS was found to be related with the concentration of sample. However, at higher sample concentrations EPS and IPS showed almost same iron chelating activities (Fig. 1f). Both EPS (66 %) and IPS (68 %) showed maximum iron chelating activity as concentration 8 mg/mL. The results are further supported by EC50 values (Table 5). EPS and IPS extracted from submerged culture of *C. cicadae* have shown significant antioxidant activities similar to *C. gracilis* [32], *C. sinensis* [49] and *C. militaris* [50]. Since antioxidants are well known for playing important roles in the human metabolic system and for protecting against cardiovascular and neurodegenerative disease, hence showing the medicinal value of submerged culture of *C. cicadae* [51, 52].

The article "Optimized extraction, composition, antioxidant and antimicrobial activities of exo and intracellular polysaccharides from submerged culture of Cordyceps cicadae" was retracted in 2018. Reasons: duplicated images; concerns about the data.

**Table 5:** EC_50_ value of EPS and IPS

Antioxidant assays	EC_50_			
	EPS (mg/mL)	IPS (mg/mL)	Ascorbic Acid	EDTA
DPPH radical scavenging activity	7*.*32 ± 0*.*00	6*.*79 ± 0*.*04	24.42 ± 2.15	-
ABTS radical scavenging activity	6*.*38 ± 0.12	5*.*23 ± 0*.*25	0.28 ± 0.02	-
Reducing power	6*.*19 ± 0*.*22	5*.*55 ± 0*.*32	0. 29 ± 0.01	-
Iron chelating activity	1*.*45 ± 0*.*32	1*.*29 ± 0*.*11	-	0.06 ± 0.0

Different letters represent the significant difference in each column and row (*p* ≤ 0.05)

Both EPS and IPS fractions showed significant antimicrobial activities against all pathogenic microorganism tested (Table 6; Table 7). The screening of antibacterial activity indicates that there were no significant differences in the power of activity between the EPS and IPS fractions. However, IPS showed slightly higher spectrum as compared to EPS. As evident from the tables, the antimicrobial spectrum was found to be directly linked with concentrations of EPS and IPS fractions. Polysaccharides from *C. cicadae* showed broad spectrum against all the pathogenic microorganisms. Maximum activities were observed against *Vibrio parahaemolyticus*. The results are similar as obtained for polysaccharides from other medicinal species of fungi [53–55]. Polysaccharides from *C. cicadae* showed activity against both gram positive and gram negative strains. The sensitivity of Gram-positive bacteria to polysaccharides extracts is in conformity with the previous studies [56, 57]. This is due to the membrane composition of the bacterial stains [58].

**Table 6:** Antibacterial activity of EPS and IPS from *C. cicadae*

Bacterial Strains	Inhibition Zone EPS (mm)				Inhibition Zone IPS (mm)				Positive control (tetra cycline)	Negative Control (EDTA)-
	25 % (con.)	50 % (con.)	75 % (con.)	100 % (con.)	25 % (con.)	50 % (con.)	75 % (con.)	100 % (con.)		
*Escherichia coli*	7.1 ± 0.5	9.2 ± 0.3	10.2 ± 0.4	11.1 ± 02	8.0 ± 0.2	10.8 ± 0.2	11.8 ± 0.9	11.9 ± 0.1	21 ± 1.52	-
*Klebsiella pneumonia*	-	-	8.2 ± 0.5	9.3 ± 0.6	-	-	8.9 ± 0.3	10.8 ± 0.3	23 ± 2.35	-
*Vivrio cholerae*	-	7.2 ± 0.2	9.3 ± 02	10.5 ± 0.8	-	7.8 ± 0.7	9.9 ± 0.2	10.9 ± 0.6	19 ± 1.50	-
*Pseudomonas aeruginosa*	8.2 ± 0.3	9.4 ± 0.6	11.3 ± 0.7	12.5 ± 0.3	8.6 ± 0.5	9.9 ± 0.5	11.5 ± 0.6	12.9 ± 0.2	18 ± 1.21	-
*Vibrio alginolyticus*	-	6.2 ± 0.8	10.5 ± 0.2	10.9 ± 0.3	-	6.8 ± 0.1	10.9 ± 0.3	11.2 ± 0.7	18 ± 2.15	-
*Staphylococcus aureus*	-	-	9.2 ± 0.8	10.1 ± 0.2	-	-	9.5 ± 0.8	10.9 ± 0.3	15 ± 2.33	-
*Vibrio parahaemolyticus*	7.3 ± 0.6	9.2 ± 0.4	10.4 ± 0.5	11.1 ± 0.9	7.6 ± 0.6	9.7 ± 0.4	10.9 ± 0.2	11.5 ± 0.8	16 ± 1.92	-
*Streptococcus pneumonia*	-	-	7.5 ± 0.1	9.2 ± 0.5	-	-	8.2 ± 0.1	9.9 ± 0.9	15 ± 1.88	-

con. – concentration, *p values* < 0.05

The article "Optimized extraction, composition, antioxidant and antimicrobial activities of exo and intracellular polysaccharides from submerged culture of Cordyceps cicadae" was retracted in 2018. Reasons: duplicated images; concerns about the data.

**Table 7:** MIC of polysaccharides extracts against tested microorganism

Species	EPS extract (mg/mL)					IPS extract (mg/mL)				
	100	80	60	40	20	100	80	60	40	20
*Escherichia coli*	++	++	+++	+++	+++	+	++	++	+++	+++
*Klebsiella pneumonia*	+	+	++	++	+++	+	++	++	++	+++
*Vivrio cholera*	+	++	+++	+++	+++	-	+	+	++	+++
*Pseudomonas aeruginosa*	-	+	++	++	+++	-	+	++	++	+++
*Vibrio alginolyticus*	-	+	++	++	+++	-	+	++	++	+++
*Staphylococcus aureus*	-	+	++	++	+++	-	+	++	++	+++
*Vibrio parahaemolyticus*	*	+	++	++	+++	+	++	++	+++	+++
*Streptococcus pneumonia*	+	+	++	++	+++	+	++	++	++	+++

*MIC concentration; − No growth; + Cloudy solution (slight growth); ++ Turbid solution (strong growth); +++ Highly turbid solution (dense growth)

Several factors are required for the production of EPS and IPS in *C. cicadae* under submerged culture condition. Factors affecting the polysaccharides production are temperature, rotation speed, pH, incubation time, carbon, nitrogen, mineral sources and carbon to nitrogen ratio. As revealed from the studies EPS and IPS exhibited excellent DPPH radical scavenging activity, ABTS radical scavenging activity, reducing power and Iron chelating activities. Present studies have revealed that the EPS and IPS of *C. cicadae* were capable to inhibit pathogenic microbes.

## Conclusion

These findings will lead the way for large scale industrial fermentations and commercial uses of EPS and IPS from *C. cicadae* as antibacterial and antioxidants constituents. Present studies will open up the scope for large scale industrial fermentation of *C. cicadae* culture for the production of biologically active polysaccharides and clinical trials of exo and intracellular on animal models Clinical trials of the polysaccharides extracted of *C. cicadae* like other commercially used *Cordyceps* species namely *C. sinensis, C. militaris* and *C. ophioglossoides, C. gracilis* etc.
